# Current Trends in Research on Bone Regeneration: A Bibliometric Analysis

**DOI:** 10.1155/2020/8787394

**Published:** 2020-05-27

**Authors:** Xin Huang, Xu Liu, Yuli Shang, Feng Qiao, Gang Chen

**Affiliations:** Department of Oral and Maxillofacial Surgery, Stomatological Hospital of Tianjin Medical University, Tianjin, China

## Abstract

**Background:**

Bone regeneration is a frequent research topic in clinical studies, but macroscopic studies on the clinical application of bone regeneration are rare. We conducted a bibliometric analysis, using international databases, to explore the clinical application and mechanism of bone regeneration, to highlight the relevant research hotspots and prospects. *Material and Methods*. Scientific reports on bone regeneration published during 2009–2019 were retrieved from PubMed. VOSviewer for cooccurrence keywords and authorship analysis. BICOMB software was used to retrieve high-frequency words and construct a text/coword matrix. The matrix was inputted into gCLUTO software, managed by biclustering analysis, in order to identify hotspots, which could achieve mountain and matrix visualizations. The matrix was also analyzed by using Ucinet 6 software for social network analysis. A strategic diagram was used for further analysis of the research hotspots of bone regeneration by “SCIMAT” software. We searched the Web of Science for relevant articles.

**Results:**

Eighty-nine high-frequency major MeSH terms were obtained from 10237 articles and were divided into 5 clusters. We generated a network visualization map, an overlay visualization mountain map, and a social network diagram. Then, the MeSH terms were subdivided into 7 categories according to each diagram; current research hotspots were identified as scaffold, drug effect, osseointegration in dental implant, guided bone regeneration, factors impacting bone regeneration, treatment of bone and tissue loss, and bone regeneration in dental implants.

**Conclusion:**

BICOMB, VOSviewer, and other bibliometric tools revealed that dental implants, scaffolds, and factors impacting bone regeneration are hot research topics, while scaffolds also hold promise from the perspective of bone tissue regeneration.

## 1. Background

Bone regeneration is necessary to address various degrees and locations of bone defects. Irrespective of whether large bone defects are caused by trauma, infection, tumor excision, and skeletal necrosis or by periodontitis, insufficient implant bone, and osteoporosis, they all require treatment involving bone regeneration. Autologous bone graft regeneration was long considered the gold standard for the treating bone defects in the clinic. However, the donor contribution is limited and the approach involves lots of complications. Additionally, this approach carries the risk of disease transmission and unsatisfactory bone integration. As an advanced technology, 3D-printed scaffolds have aroused wide concern over the past few decades due to their unique physical properties for tissue regeneration engineering and vascularized bone regeneration [1, 2].

Periodontal disease, which can lead to damage of the periodontal ligament and alveolar bone, is a common oral health problem in the elderly population and is prevalent in an aging society [3]. Treatment of periodontitis is aimed at preventing further disease progression and, if possible, at restoring lost periodontal and bone tissues in order to support patients in maintaining oral health [4]. Hence, bone regeneration is an excellent treatment approach for periodontal disease.

In another respect, dental implants for the elderly should be designed as easy maintenance prostheses or removed. It could be a policy to promote oral health and comfort in the final stage of life [5]. Dental implants and bone regeneration fields have always been intertwined. Various lines of evidence have demonstrated that guided bone regeneration could successfully provide missing bone at implant sites with insufficient bone volume [6]. Increasingly, studies have advocated the concept of early implantation and immediate implantation, which offers superior soft tissue stability and preserved horizontal ridge dimension and buccal plate thickness [7, 8]. The continuous development of nanotechnology has led to faster bone formation, reduced healing time, and rapid recovery to function with new implants [9]. Additionally, as a future trend in the field of oral medicine, digitization is increasingly used in oral surgery. For example, dental implant surgery can now be guided by cone-beam computed tomography and digital guide plates, which could improve clinical experiences and superior evidence-based outcomes, offering clinicians more confidence and markedly more convenience to patients [10, 11].

Bone regeneration is a complicated physiological process involving histological and biological changes, associated with blood supply, inflammation, and the formation of fibrous tissue and bony callus, which are constitutionally induced by both local and recruited cells. In the last few years, numerous studies have confirmed that various bone growth factors, such as bone morphogenetic protein (BMP), transforming growth factor *β* (TGF-*β*), insulin-like growth factor (IGF), and platelet-derived growth factor (PDGF), play momentous roles in the process of bone regeneration. In particular, BMPs, including BMP-2, make a critical difference in the differentiation of osteogenic progenitor cells into osteoblasts and in the bone mineralization process [12]. However, the optimal dosage of BMP-2 to be used in bone regeneration has not been determined to date [13]. To address this issue, drug delivery systems have been employed, in which drugs are incorporated into and released by biomaterial carriers [14]. In more recent studies, dual-controlled drug release, in which two drugs with different biological effects are released to induce synergistic bone regeneration, has offered an even more attractive strategy [15].

Although there have been various systematic reviews on the application of and mechanism underlying bone regeneration during the past 10 years [7, 8, 16], no macroscopic overview of bone regeneration has been reported. Such an overview could guide further research based on the hotspots for development and tendency in the application of and mechanism underlying bone regeneration.

In the literature review of bone regeneration, scientists may merely explore topics or literature in a single direction, in which case, however, the content of exploration will be narrow. Hence, we use a variety of tools to comprehensively analyze the status of bone regeneration studies through bibliometric analysis. Furthermore, the future and current research hotspots of the research theme of bone regeneration were revealed from multiple perspectives, and the key research directions in this field were determined. By focusing on bone regeneration, we are able to construct a general analysis of bibliometric effective models, which can help identify and evaluate achievements in the field to guide experimentation strategies and funding decisions.

Bibliometrics, a well-established research method in information science, has been demonstrated to be an effective tool to research a subject's status [17]. We performed a bibliometric analysis, using international databases, to explore the application and mechanism of bone regeneration in clinical practice and identify hotspots in a research field. In bibliometrics, the coword analysis first invented by French bibliographers is frequently used to definite research hotspots. We consider that if two terms appear in the same article concurrently, it means that they may have a potential relationship. Further, in the same article, if these two terms appear frequently at the same time, they are considered to be closely related. After some analysis of these cooccurrence relations such as cluster analysis or factor analysis, keywords that reach the threshold are considered as a hot topic in this research area [18]. Cluster analysis is the basis for obtaining semantic relationships of related research theme. Compared with traditional cluster analysis, biclustering analysis on the subject words can be performed with the rows as well as the columns being clustered simultaneously in the matrix [19]. It can also execute cluster analysis on the entire information or part of a large amount of data [20].

Due to the abstract nature of the target text information in bibliometrics, visualization tools, such as BICOMB, Ucinet 6, gCLUTO, SCIMAT, and VOSviewer, are necessary for bibliometric analysis, for example, using BICOMB to analyze the hotspots of the topic of bone regeneration through coword analysis, using VOSviewer to analyze the strength of links between journals and the connections between authors [21], and using SCIMAT to analyze the bibliometric characteristics of bone regeneration and predict the future development potential.

In addition, altmetrics are used as a method to quantify the social media attention and comments received by scientific work. It is a supplement and assistance to bibliometrics. We believe that it has a great potential for evaluating research impact [22].

In this article, all research directions related to the dental implants, scaffolds, and factors impacting bone regeneration were considered to provide novel insights into study on the bone regeneration over the past 10 years.

## 2. Material and Methods

### 2.1. Data Resource

PubMed is a database of biomedical papers and abstracts; although its core theme is medicine, it also includes other areas related to medicine. The search engine is provided by the National Library of the United States as part of the Entrez Information Retrieval System. We searched PubMed using the following search strategy: “Bone Regeneration”[Mesh] AND (“2009/08/01”[PDAT]: “2019/07/31”[PDAT]).

The titles and conclusion of publications identified using this strategy were then screened based on interarticle correlation and selection criteria. We included papers when their contents primarily focused on bone regeneration and its application and underlying mechanism, and articles were excluded if they involved animal studies or science briefings.

Subsequently, 2 researchers (Xin Huang and Xu Liu) independently assessed and studied each of the 10823 identified papers and reached a consensus on inclusion of the paper for analysis. Two investigators came to an agreement of 96% (kappa = (*P*_0_ − *P*_e_)/(*n* − *P*_e_) = 0.96 > 0.75), which indicated a high consistency [23]. Consequently, a total of 10237 articles were selected in this study.

For each article, the following key items were downloaded from PubMed: title, authors, institution, country, source, year, and MeSH terms. The collected data were saved in XML and MEDLINE formats.

### 2.2. Information Extraction and Coword Analysis

The research used Bibliographic Item Co-Occurrence Matrix Builder (BICOMB) to perform data extraction and matrix construction. A cooccurrence matrix can be generated by this software, and the matrix can be used as basic data for following analysis. BICOMB was designed by Professor Lei Cui from China Medical University and was furthered upgraded to version 2.0 under funding from the China Medical University [17].

After coword analysis, a coword matrix was created by BICOMB and then input into Ucinet 6 software, which was designed by Stephen Borgatti and colleagues from the University of California, Irvine, for social network analysis (SNA). All the major MeSH terms with high frequency were visualized after extracting data to explore research hotspots for bone regeneration. It was possible to reveal the connection between major MeSH terms and high-frequency source references by referring to biclustering.

Subsequently, we use the gCLUTO version 1.0 software, which was a graphical cluster toolkit and designed by Rasmussen and Karypis of Minnesota University [24], to take advantage of the binary matrix constructed from BICOMB for further analysis. In this matrix, the content of the row was the MeSH term frequency and the column was PMID of original article. The double cluster parameters in gCLUTO are set according to the parameters suitable for biclustering analysis [25]. The clustering method chooses repeated bisection, cosine was set to the similarity function, and I2 was set to the clustering criterion function.

To determine the best numbers of clusters, we repeated the search by using different numbers of clusters to obtain the minimum and ideal external similarity (ESim) and internal similarity (ISim). We obtained high-frequency dual-focus results with MeSH articles by generating a visualized mountain map. Utilizing the semantic relationship between MeSH terms and the research purposes of representative papers in each group, the basic direction of bone regeneration hotspots and their applications were abstracted and analyzed.

Meanwhile, VOSviewer generated a network visualization map based on high-frequency keywords. And it generated an overlay visualization map based on the connection of the author of the journal.

In order to describe the hot topic distribution in the area of bone regeneration, we used the carrot system to search for articles; this is an online visualization system based on PubMed. Then, a strategic diagram was used for further analysis of the research hotspots of bone regeneration, by implementing SCIMAT software. We searched the Web of Science (WOS) for relevant articles and obtained articles about bone regeneration published from Jan 1, 2010, to Sep 30, 2019. The strategic diagram implements 2-dimension coordinates, employing centrality and density as parameters to construct a diagram describing the internal integrity of certain categories and their interacting influence with other disciplines [26]. In the strategic diagram, the intensity of the interacting influence is presented with the *x*-axis which is set as centrality. We found that the centrality of the sort is determined by the tightness of the links between the main areas of the sort and other sorts [27]. The internal relationships within particular sorts are presented with the *y*-axis which is set as density. It represents the potential for future development. The average links within a sort determine the density of a sort.

## 3. Results

### 3.1. Bone Regeneration Research Hotspots

Bone regeneration research hotspots among publications from Aug 1, 2009, to Jul 31, 2019, revealed 6673 major MeSH terms. We define 24645 high-frequency major MeSH terms as occurred more than 100 times through our publication analysis. According to the BICOMB analysis consequence, which is previously described, we take high-frequency main MeSH term matrix as row labels and the source articles as column labels. The matrix (localized view shown in Table 1) demonstrates the validity of the main MeSH terms in the source article. The “1” in the cell means high-frequency major MeSH terms occur in this article, and the “0” means there are none.

Cooccurrence of terms in the publications reveals the relevance of the research purposes (Table 2), and the keyword network generated by matrix is associated with the knowledge structure [28]. The network graph is illustrated in Figure 1, which indicates the overall structure of bone regeneration research. Both the subsection of the research and the degrees of correlation among keywords are represented. For each node, the more cooccurring frequencies, the larger the node area. This keyword is the core of bone regeneration research, such as dental implant, osseointegration, tissue scaffolds, and titanium. Red links are tighter than green links, indicating a higher frequency of cooccurrence. Thick lines make connections between bone regeneration and tissue scaffolds, dental implants, and osseointegration, which indicate that these keywords are of vital importance in nowadays research.

Various clusters were used in biclustering analysis. The biclustering results for the high-frequency main MeSH term source matrix are shown in the mountain and matrix visualizations.  Figure 2 shows each cluster represented as a peak, labeled by cluster numbers 0–4. The altitude, volume, and color of the peaks are applied to depict information about the related clusters. The peak shows the position of the cluster on the plane relative to that of other clusters. The distance between the peaks in one plane indicates the relative similarity of corresponding clusters. The height of the peak is proportional to the potential correlation among the clusters directly. The volume of the peak is relative to the number of major MeSH terms with high frequency containing in one cluster. The internal standard deviation of a clustered object was represented by the color of peak, the red part of the mountain means low, and the blue part means high. The descriptive and discriminating features of articles in each cluster are shown in Table 3.

Moreover, some clusters may be subdivided into narrower topics based on the following standards, as determined by discussion within the study group: (1) the semantic connection between the MeSH vocabulary and a larger cluster; (2) the category of the MeSH terms. Accordingly, each narrower topic was concluded to 7 hotspots, respectively, which were found in the area of bone regeneration: (1) the drug effects and pharmacological studies on bone regeneration (cluster 0); (2) the connection between dental materials and osseointegration in dental implants (cluster 1); (3) the materials and methods involved in guided bone regeneration (GBR) (cluster 2); (4) scaffold (cluster 2); (5) physiological, cytological, and histological factors influencing bone regeneration (cluster 3); (6) treatment of bone and tissue loss caused by periodontitis (cluster 4); and (7) dental implants and the methods of resolving the issue of insufficient implant bone (cluster 4).

In the network visualization map (Figure 3), items are represented by circles. The larger the circle, the heavier weight the item. However, for some duplicate items, the label may not be displayed. Items in different clusters have different colors. The lines between items represent links. The distance reflects the relevance of the journal, such as biomaterials and scaffolds, mesenchymal stem cells and stem cells, drug delivery, and bone tissue engineering. If the lines are thick, it will mean strong links between journals.

In the overlay visualization map of authorship (Figure 4), if two or more authors are cited by one or more subsequent articles at the same time, it is said that these two or more authors constitute a cocitation relationship. The author is represented by the node, the color of the node is determined by the average time of each key year. For example, the article “chang, jiang” appears twice in 2014 and four times in 2016; then, the color appears in the color indicated by ((2014∗2 + 2016∗4)/2 = 2015.3). For those authors who have high influence in the field, the node has a larger area, for example, Miron, Richard J, Chang, Jiang and Reis, and Rui. If the author has a multidisciplinary background or the research field has interdisciplinary attributes, the node connects to two or more nodes.

In the carrot diagram, the area of each grid represents the frequency of occurrence of these keywords (Figure 5). Thus, we found that dental implants, bone repair, bone grafting, tissue engineering, scaffolds for bone and tissue, membrane, and osteogenic differentiation were hotspots in bone regeneration. Moreover, there was a close connection between these keywords, such as between periodontal regeneration and mesenchymal stem cells (MSCS) [29], and bone repair, BMP, and bone grafting [30]. Furthermore, even if these keywords had no direct connection in Figure 1, these factors would be connected with each other in a clinical context, for example, GBR and membranes [31, 32].

In strategic diagrams, all the spheres of 4 quadrants represent different themes, and the location of different quadrants were determined by their internal and external cohesion, which separately indicated density and centrality. As demonstrated in Figure 6, the area of the spheres is relative to the number of MeSH terms with high frequency. Hotspots and cores of those studies have both strong centrality and high density, as shown in Quadrant 1 (upper-right), which represents that those themes have a high degree of foresightedness and receive marked attention. The content of studies in Quadrant 2 (upper-left) is supposed to those topics currently less-well researched, receiving less attention, but which represent a potential area of research. Quadrant III (lower-left) contains themes with a low degree of novelty and attention; these research topics are outdated and do not fit the current trend. The last quadrant, Quadrant IV (lower-right), contains themes receiving a high degree of attention, but which are not trending and are not the up-and-coming research focus. Scaffold, factors impacting bone regeneration, and materials and applications related to dental implant were located in Quadrant I, representing that those themes have a core status, with high density and centrality. This was in accordance with the results of the visualized mountain map, matrix, SNA, and carrot diagram. The research topics in Quadrant III were in relatively remote, “cold” fields.

## 4. Discussion

With the continuous development of regenerative medicine, the number of research literature and journals on bone regeneration is also growing rapidly. In this study, we used various bibliometric tools to study the literature on bone regeneration in the last ten years in order to determine which areas are the focus of bone regeneration research and which areas have more potential and prospects. This will provide researchers with more accurate research directions. More importantly, the results of bibliometrics research should be used not only to assist in making decisions about research funding but also to help companies choose more promising R&D directions.

BICOMB is used for MeSH term extraction and cooccurrence matrix generation, and gCLUTO performs biclustering analysis. In the mountain peak graph (Figure 2), we obtained 5 main clusters, which are further divided into 7 main topics (later in this article). We will analyze these 7 topics in detail. These 7 topics are considered to be the hotspots of bone regeneration research. VOSviewer is used to generate a network visualization map and an overlay visualization map of authorship. In the network visualization of keywords related to bone regeneration, we identified key keywords: scaffolds, mesenchymal stem cells, osteogenic differentiation, and dental implant. These keywords will be used as hotspots in bone regeneration research, providing researchers and scientists with topical directions. Researchers have found high-impact authors about bone regeneration through overlay visualization of authorship.

SCIMAT is used to generate strategic coordinate diagrams. Keywords in the first quadrant such as dental implant, survival, prostheses, and titanium have higher attention and maturity. Keywords in the fourth quadrant such as immediate-loading and marginal-bone-loss have higher attention, but the maturity is insufficient. We believe that with the continuous improvement of technology, it will become a new hotspot in the future.

In this study, different bibliometric tools generate diverse diagrams to analyze the literature of bone regeneration. For example, carrot diagram is simple to make and can intuitively represent the hotspot distribution and connection of bone regeneration. However, carrot diagram is not as accurate as strategic coordinate diagram. On the one hand, the production of strategic coordinate diagram is complicated, whose data format needs to be transformed. Furthermore, producing cooccurrence matrices and calculating density, centripetalism is very tedious. On the other hand, it can show the core points of this research field most intuitively, technology maturity, development potential, and popularity trends for reader. Compared with the above literature metrology tools, VOSviewer is a free software based on JAVA, which is easy to download and easy to operate. And it can generate 3 kinds of visualization at the same time. Its map themes and connections are clear. But for data, it requires operator screening, data cleaning, and format conversion, which are more time consuming.

BMPs hold great promise for the fields of bioengineering and regenerative medicine. BMP-2 is commonly used to induce bone regeneration, and studies have shown that BMP-2 could enhance bone repair and bone regeneration [33]. However, the optimal dosage of BMP-2 for bone regeneration has not been determined to date [13]. In recent studies, attempts have been made to find the appropriate dose that would optimize bone regeneration and minimize adverse effects of high-dose BMP-2 therapy [34]. Other studies, such as the effects of blood extracts, including concentrated growth factors and platelet-rich fibrin or statins on bone formation, are also the focus of current clinical and fundamental research, which can prove the importance of drug effects on bone formation.

Stem and progenitor cells contributed to bone repair/regeneration [35]. Due to the significant role played by MSCS in bone regeneration, understanding the molecular signaling pathways associated with MSCS may be important for the development of bone implants, bone substitute materials, and cell-based scaffolds for bone regeneration [36].

At the moment, hydroxyapatite (HA) has been widespread investigated for biomedical use mainly due to the similarity composition as bone. The microstructure, stability, and crystallinity of the HA structure in an implant can be altered by a microsubstituent. And some experimental investigations have shown that the substituent can also have a remarkable effect on bone cells combining the implant. As a consequence, it can facilitate the new bone formation and bone remodeling procedures [37]. A recent study has shown that different metal ions are integral components of bone tissue. Furthermore, it has been revealed that the concentration of the released metal ions plays a vital role in the bone formation process [38].

As one of the hotspots and cores of studies in the area of bone regeneration in recent years, scaffolds are widely used in bone regeneration. In the clinic, in order to overcome the limitations of bone grafts or implants, tissue engineering of 3D scaffolds plays a very important role [39]. An analysis of existing scaffold materials showed that use of scaffolds could improve bone formation in oral regenerative therapy [40]. In addition, poly(fumaroyl bioxirane) maleate (PFM), a newly developed functional polymer with numerous functional groups, could serve as a promising and effective optimization method for traditional scaffolds in bone regeneration [41]. Thus, scaffolds are an important option for bone tissue regeneration. A large number of reports and clinical trials have proven that scaffold use is a necessary factor for promoting osteogenesis; this was also confirmed in the mountain and matrix visualizations, social network diagrams, and strategic diagrams produced in this study. It is particularly noteworthy that the combination of scaffold and drugs is also a hot topic of relevant research.

Treatment of insufficient bone mass in the implant area is a common issue faced by oral surgeons. In the maxillary molar area, especially when the distance between the maxillary sinus and the alveolar ridge is too small, and when there is insufficient bone tissue to support the implant, sinus elevation is generally used to resolve the problem of insufficient bone mass. For alveolar defects in local regions of the jaw, GBR is widely used [6]. In other respects, for large bone defects caused by trauma, infection, tumor excision, and skeletal necrosis, the common and effective repair method is bone transplantation. In a word, in the field of oral implants, especially in terms of esthetics, there are often cases of bone defects or insufficient bone mass requiring bone grafting, and it is usually necessary to combine GBR technology and implant osteogenic scaffolds to achieve the purpose of implant osseointegration, which is consistent with the results of this study.

Periodontal disease, which can lead to destruction of the periodontal ligament and alveolar bone, is a common oral health problem [3]. The final goals of periodontal treatment are the complete regeneration of alveolar bone loss to the destructive inflammatory immune response, or to trauma, with tissues that possess the same structure and function. And it can be attempted to reestablish a sustainable health-promoting biofilm to take the place of the dysbiosis [42]. In order to find an optimal solution, a series of different surgical techniques is used in general, often including implantation of diversified types of bone graft and/or bone substitutes like bioss, root surface demineralization, guided tissue regeneration, and utilization of growth and differentiation factors, in order to achieve tissue and bone regeneration [43].

At present, an important indicator for the success of oral implantation is osseointegration; the biocompatibility of dental implant materials is significant for the formation of implant osseointegration. With the development of nanotechnology, a great many researches have indicated that the application of nanoparticles as implant-coating materials can improve the implant success rate and improve soft tissue integration and osteogeneration [44]. Moreover, many studies have found that the implant success rate can also be improved through implant surface modification [45].

Biofilms made from biomaterials can artificially erect a biological barrier between the soft tissues of the gums and the bone defects and guide complete bone repair in the bone defect area, in the GBR approach. This is among the most important technologies for implant surgery today. Various studies have confirmed that implant placement with simultaneous contour augmentation through GBR, using a 2-layer composite graft in postextraction single-tooth sites, could provide stable bone conditions [46]. However, the application of GBR also has negative side effects that increased the time of treatment and healing and increased the costs to patients with greater morbidity [47]. In recent studies, a new bilayer membrane was developed for GBR, and the biocompatibility and potential applicability of these membranes for GBR treatment have been confirmed [48]. Furthermore, GBR technology not only guides the regeneration of bone defects but also increases bone mass and increases the height and width of local alveolar ridges in the implant targeted area.

Although traditional bibliometric analysis is considered a standard method for evaluating “journals, authors, and research institutions,” we can only study published journals. For some meaningful data, it is very likely to “lost.” But using social media tools may reduce this situation [22].

With the continuous popularity of social media, people's access to scientific information has fundamentally changed. As a tool to quantify the social media attention received by scientific work, altmetrics have attracted the attention of researchers. As a supplement to bibliometric tools, it has a great potential for researching impact [49]. Just as Bornmann believes, height measurement data should not only be used to make decisions about research funding but also be used to assist rather than replace bibliometrics. Overall, the indicator should not outperform peer review but should supplement it [50].

However, there are still some limitations in this study. Because collaborative cluster analysis of high-frequency MeSH terms is a new analysis method, researchers will have a certain degree of bias when selecting vocabulary. Due to functional limitations in the PubMed and Web of Science databases lacking other database retrieval results, the data set in this study may be incomplete. In addition, due to the inconsistent quality of articles, errors in some research results are inevitable. At present, the visualization software we use, such as Ucinet 6, VOSviewer, SCIMAT, and other processing documents, often can only process one database in one time, which has limitations of biased results. The results of analyzing multiple databases will be more objective and accurate.

## 5. Conclusion

Biclustering analysis depicted the connection between the application and the research of bone regeneration. In this study, we generalized 3 directions and 7 hotspots of bone regeneration research. We found that there is a close association among bone regeneration, dental implants, and factors impacting bone regeneration. Bone regeneration is an important consideration in the treatment of certain diseases, especially periodontal disease. The study and application of scaffolds have a great potential value in the future. In conclusion, we can use these methods to understand the research hotspots and prospects of bone regeneration from a macroscopic view, which can make it easier for researchers to master future research trends, facilitating clinical and fundamental research.

## Figures and Tables

**Figure 1:** Social network analysis (SNA) of top 30 MeSH terms with high frequency related to bone regeneration studies, published during 2009–2019. The keyword's centrality is presented by the size of nodes, and the cooccurrence frequency of keyword pairs is presented by the thickness of the lines.

**Figure 2:** A visualized mountain map biclustering of major MeSH terms with high frequency and articles on bone regeneration.

**Figure 3:** Network visualization map of keyword.

**Figure 4:** Overlay visualization map of authorship.

**Figure 5:** A survey of major topics in bone regeneration. The visualizations were obtained using the carrot system, based on the top-ranking results of the search.

**Figure 6:** A strategic diagram based on reports involving bone regeneration published from 2010 to 2019.

**Table 1:** High-frequency major MeSH term source article matrix (localized).

No.	Major MeSH terms	PMIDs of source article				
		18508337	18523038	18523954	…	31352944
1	Dental implants	0	0	0	…	0
2	Bone regeneration	0	0	0	…	0
3	Bone regeneration/drug effects	0	0	0	…	0
…	…	…	…	…	…	…
89	Calcium phosphates/therapeutic use	0	0	0	…	0

**Table 2:** A coword matrix of major MeSH terms with high frequency (localized).

No.	Major MeSH terms	Dental implants	Bone regeneration		Calcium phosphates/therapeutic use
1	Dental implants	1673	41	…	6
2	Bone regeneration	41	1579	…	0
3	Bone regeneration/drug effects	23	0	…	0
…	…	…	…	…	…
89	Calcium phosphates/therapeutic use	5	16	…	101

**Table 3:** Descriptive and discriminating features of each cluster.

Descriptive and discriminating features				
Cluster 0	Size 13	ISim:0.132	ESim:0.016	
Descriptive	29931022	29532542	25769221	25916272
Discriminating	29931022	29532542	25769221	25675839
Cluster 1	Size 18	ISim:0.114	ESim:0.013	
Descriptive	27405685	24664938	19615586	25860058
Discriminating	27405685	19615586	25860058	21441047
Cluster 2	Size 18	ISim:0.114	ESim:0.017	
Descriptive	27427599	22509754	21658081	23611676
Discriminating	27427599	24692259	29025652	22427485
Cluster 3	Size 18	ISim:0.106	ESim:0.016	
Descriptive	30865107	22627404	29027958	23359411
Discriminating	30865107	22627404	29027958	23359411
Cluster 4	Size 22	ISim:0.092	ESim:0.011	
Descriptive	25106010	20831755	23057053	24179978
Discriminating	25106010	23057053	24179978	20491837

## Data Availability

All the data cited in this paper were quoted from PubMed and Web of Science databases.
